The article "Changes in Nutritional Status of Cancer Patients Undergoing Proton Radiation Therapy Based on Real-World Data" was published in 2023. Journal: J Healthc Eng.

# Changes in Nutritional Status of Cancer Patients Undergoing Proton Radiation Therapy Based on Real-World Data

**DOI:** 10.1155/2023/9260747

**Published:** 2023-02-14

**Authors:** Menglin Wang, Yue Zhu, Yinghui Ju, Tengfei Long, Lingtai Jin, Jin Zhang, Yangyu Zhao, Honglian Wang, Rui Wu

**Affiliations:** ^1^Hefei Ion Medical Center, The First Affiliated Hospital of USTC, Division of Life Sciences and Medicine, University of Science and Technology of China, Hefei, China; ^2^Department of Pharmacy, The First Affiliated Hospital of USTC, Division of Life Sciences and Medicine, University of Science and Technology of China, Hefei, China; ^3^Department of Pharmacy, The People's Hospital of Huangshan, Huangshan, China

## Abstract

**Methods:**

Observational study on 47 adult hospitalized cancer patients including 27 males and 20 females who received proton beam radiotherapy during December 2021 and August 2022. Nutritional assessments, 24 h dietary survey, handgrip strength (HGS) test, anthropometrical measurements, and hematological parameters were conducted or collected at the beginning and the completion of treatment.

**Results:**

The rate of nutritional risk and malnutrition among the total of 47 enrolled patients was 4.3% and 12.8% at the onset of proton radiation and raised up to 6.4% and 27.7% at the end of the treatment. 42.6% of patients experienced weight loss during the proton radiotherapy, and 1 of them had weight loss over 5%, and in general, the average body weight was stable over radiotherapy. The changes in patients' 24 h dietary intakes, HGS, and anthropometrical parameters, including triceps skinfold thickness (TSF), midupper arm circumference (MUAC), and midupper arm muscle circumference (MAMC), were statistically insignificant over the treatment (all *p* values > 0.05). The changes in patients' hematological parameters, including total protein (TP) and serum albumin (ALB), were not statistically significant over the treatment (all *p* values >0.05), and the level of hemoglobin (HGB) at the end of treatment was higher than that at the onset (*p* < 0.05).

**Conclusion:**

The results of this study demonstrated that proton radiotherapy might have a lighter effect on the nutritional status of cancer patients.

## 1. Introduction

Nearly 19.3 million new cancer cases and over 9.9 million deaths were reported worldwide in 2020 [1]. Malnutrition is a common problem in cancer patients, and a range from 20% to 80% of oncology patients suffered from different degrees of malnutrition during their illness, which was closely associated with tumor type, location, stage, and therapies [2, 3]. Previous studies suggested that poor nutritional status has a negative impact on patients by reducing the effectivity and tolerance of treatment, quality of life, and clinical outcome and increasing the risk of complications, infections, and healthcare costs [4–6].

On the other hand, malnutrition can be aggravated by treatment-related complications. Antitumor therapies, including chemotherapy and radiotherapy, are often accompanied by many adverse reactions [6]. Radiotherapy can induce various nutrition impact toxicities such as dysphagia, xerostomia, oral mucositis, and enteritis, which are correlated with location, and may worsen patient's nutritional status by reducing oral intakes or nutrition absorption [7–9]. Unsal et al. [10] showed that the prevalence of malnutrition in cancer patients was raised from 31% up to 43% at the end of radiotherapy.

Proton radiotherapy (PRT) is a technological advanced radiotherapy with a characteristic Bragg peak which deposits the maximum dose at a specific depth and no exit dose in normal tissues [11, 12]. It now has been accepted in treating esophageal cancer, head and neck malignancies, and many other cancers [13–15]. Compared to conventional photon therapy, proton therapy has advantages in improving patients' clinical outcomes including the improvement of overall survival and the reduction of adverse effects [12, 16–19].

Despite the advantages of proton therapy, adverse effects such as fatigue, and weight loss were also reported [20]. Weight loss is a common symptom of malnutrition. Hebuterne et al. [2] reported that 84% of the cancer patients had experienced weight loss, and 51% of them had lost more than 5% of their body weight since disease onset. Among patients who received proton radiation, 58.72% had weight loss during their treatment [21]. However, there are rare investigations on the nutritional status of cancer patients undergoing proton therapy. In this present study, we evaluated the nutritional status of cancer patients over proton radiation and aimed to investigate the effect of PRT on nutritional status of cancer patients.

## 2. Methods

### 2.1. Participations

This observational study was carried out in Hefei Ion Medical Center (HIMC) in Hefei, China, from December 2021 to August 2022. All patients with definite pathological diagnosis of cancer were asked if they received proton beam radiation therapy at HIMC. Inclusion criteria were as follows: (1) age ≥18 years. (2) A pathological diagnosis of cancer. (3) Complete proton radiation. (4) Conscious and no communication disorders. (5) Willing and able to give their informed consent. (6) Able to complete the process of nutritional screening and assessment and cooperate with physical measurement. This is an observational study, and no intervention was taken during the study period, and registration number is not applicable.

### 2.2. Data Collection

Patient clinical information such as age, gender, tumor morphological type, TNM stage, radiotherapy strategy, and hematological parameters were obtained from medical records. NRS-2002, PG SGA, 24 h dietary survey, handgrip strength (HGS) test, and anthropometrical measurements were conducted separately at the beginning and the end of proton treatment.

### 2.3. Nutritional Risk Assessment

Nutritional Risk Screening 2002 (NRS 2002) was used to assess malnutrition risk. It is a nutritional risk screening tool which was proposed by Kondrup et al. [22] based on 128 randomized trials. It was verified and widely used in many studies [5, 23–25], and now is recommended by the European Society for Parenteral and Enteral Nutrition (ESPEN), Chinese Society of Parenteral and Enteral Nutrition (CSPEN), and many other guidelines [26–28]. NRS 2002 including three parts [22]: impaired nutritional status (0∼3), severity of disease (0∼3), and age score (70 years or over has 1 score). The sum of score is 0∼7, a score of 3 or higher indicates that there is a nutritional risk, and scores of less than 3 can be considered as no nutritional risk.

### 2.4. Nutritional Status Assessment

Patient Generated Subjective Global Assessment (PG SGA) was first proposed by Ottery FD [29] in 1994, which was especially suitable for the nutritional assessment of cancer patients. It consists of two sections: (1) the patient-completed section which including four aspects: weight loss, food intake, nutritional impact symptoms (NIS), and functional capacity, (2) the clinician-completed component which assesses three aspects: disease and age, metabolic stress, and physical examination. Based on these assessments, patients are classified as PG SGA A (0∼3), B (4∼8), or C (≥9), which was represented as well nourished, moderately or suspected of being malnourished and severely malnourished.

### 2.5. Dietary Survey

24 h dietary intake including food type and quantity was recorded to estimate the amount of daily energy and protein intake.

### 2.6. Handgrip Strength

Handgrip strength test in a non-dominant hand or no-injured hand was referenced to Santos et al. [30] and performed by using an electronic hand dynamometer (EH101, Zhongshan Camry Electronic Co. Ltd., Zhongshan, China) with a resolution of 0.1 kg. HGS <26 kg for men and <18 kg for women was considered as low handgrip strength (LHS) according to the Asian Working Group for Sarcopenia (AWGS) recommended in 2014 [31].

### 2.7. Anthropometry

Anthropometrical measurements including weight, height, body mass index (BMI), triceps skinfold thickness (TSF), mid-upper arm circumference (MUAC) and mid-upper arm muscle circumference (MAMC) were collected. BMI was calculated as weight (kg) divided by height squared (m^2^). MUAC was obtained by using a tape measure with a resolution of 0.1 cm. TSF was obtained by using a fat-thickness measure (TiXing, Changshu Xinfeng Instrument Co. LTD., Suzhou, China) with a resolution of 0.5 mm. TSF, and MUAC were repeated 3 times each time, and average values were taken. MACM was calculated by performing the formula: MAMC (mm) = MUAC (mm) − *π* × TSF (mm).

### 2.8. Hematological Parameter

Patients' laboratory data at the onset and the end of proton treatment were collected, which including total protein (TP), serum albumin (ALB), and hemoglobin (HGB).

### 2.9. Quality Control

All investigators were trained to conduct nutritional assessments and anthropometric measurements, and at least two investigators participated in each assessment and measurement. Data were settled and inputted by one investigator and checked by two other investigators. After confirmation, data were used for statistical analysis and were unable to change.

### 2.10. Statistical Analysis

IBM SPSS Statistics 25.0 software (IBM, Armonk, US) was used for performing statistical analysis. Continuous variables were expressed as mean ± standard deviation (SD) or median and interquartile range (IQR), and categorical variables were expressed as number and percentage. The comparison of continuous variables between groups was performed by the paired *t* -test if they were normally distributed, otherwise, the Wilcoxon signed rank sum test was carried out. The comparison of categorical variables between groups was performed by Pearson's *χ*^2^ test or Fisher's exact test. All tests were two-side and *p* < 0.05 was considered statistically significant.

## 3. Results

### 3.1. Patients

A total of 47 hospitalized patients received PRT and completed our investigations from December 2021 to August 2022. The demographic and clinical characteristics of enrolled patients are shown in Table 1. Of all participants, 27 were males, and the range of patients' age was from 26 to 76 years, with the median age was 55 years. The median patients' body weight was 65 kg, with a range from 42 to 99 kg. 12 (25.5%) patients with head and neck cancer, 13 (27.7%) patients with intracranial tumor, 6 (12.8%) patients with lung or chest cancer, 16 (34.0%) patients with abdomen, pelvis, and other cancers.

### 3.2. Nutritional Assessments

Nutritional assessments were conducted at the onset and the end of PRT. According to NRS 2002 assessment, scored 3 or greater were defined as nutritional risk, 2 (4.3%) patients with nutritional risk at the onset of PRT, and 3 (6.4%) patients at the end of PRT, the proportion of nutritional risk showed no significant difference between before and after PRT (*p* > 0.05, Table 2).

According to PG SGA assessment, patients are classified as well nourished (PG SGA A, 0∼3), moderate malnourished (PG SGA B, 4∼8) and severe malnourished (PG SGA C, ≥9). At the onset of PRT, 6 (12.8%) patients were moderate malnourished, while in the end of PRT, 11 (23.4%) patients were moderate malnourished and 2 (4.3%) patients were severe malnourished (Table 2, *p* > 0.05). The rate of malnutrition assessed by PG SGA was 12.8% initially and raised up to 27.7% at the end of PRT (Table 2). But the proportion of malnutrition showed no significant differences at the onset and the end of PRT (*p* > 0.05, Table 2).

The median percentage of the change in patients' weight during PRT was 0.00% (range from−5.3% to 9.2%). 20 (42.6%) patients experienced weight loss during PRT, only 1 (2.1%) patient had over 5% weight loss, 12 (25.5%) patients maintained their body weight over treatment, 15 (31.9%) patients gained their weight during PRT, and 2 of them had over 5% weight gain (Table 2).

According to BMI (Table 2), none of the 47 patients were underweight at the onset and the end of treatment, and there was no change in the proportion of underweight, normal weight, overweight and obese (*p*=1) according to BMI cut-off points for Asian populations recommended by WHO [32].

### 3.3. Dietary Survey

According to the dietary survey, the average of patients' daily energy intake was lower at the end of treatment than at the onset, but the difference was insignificant (*p* > 0.05, Table 3). The daily protein intake showed no significant change between onset and the end of PRT (*p* > 0.05, Table 3).

### 3.4. Handgrip Strength

The average strength of non-dominant hand or no-injured hand was 31.35 ± 10.06 kg at the onset and 30.16 ± 9.87 kg at the end of treatment, 6 (12.7%) patients at onset and 5 (10.6%) patients at the end of PRT were LHS, but these changes in HGS were insignificant (*p* > 0.05, Table 4).

### 3.5. Anthropometry

There were no significant differences were observed in PRT received patients' weight, BMI, MUAC, MAMC, and TSF between the onset and the end of their treatments (all *p* values > 0.05, Table 5).

### 3.6. Hematological Parameter

At the onset of treatment, 1 of the 47 patients did not have TP and ALB detected. As shown in Table 6, no significant difference was observed in the levels of total protein and albumin between the beginning and the completion of PRT (all *p* > 0.05, Table 6). The levels of patients' hemoglobin at the end of PRT were higher than those before PRT (*p* < 0.05, Table 6).

## 4. Discussion

Patients with cancer were at high risk of malnutrition, the prevalence of malnutrition varied with primary tumor type, location, and stage. Previous studies have evaluated that 20∼80% of oncology patients suffered from malnutrition, of common malignant tumors, pancreatic, esophageal, gastric cancer, head and neck, and lung cancer had a higher risk of malnutrition [2, 33]. Poor nutritional status increased the risk of an unplanned treatment break and had a negative effect on clinical outcomes [4, 6]. Furthermore, patients' nutritional status can also be exacerbated by antitumor treatments including radiation. An investigation of Unsal et al. [10] showed that malnutrition was present in 31% of conventional radiotherapy received patients at the onset of treatment and 43% at the end of treatment. Hill et al. [6] reported that 63.6% of gastrointestinal cancer patients were well-nourished at baseline and that figure was reversed to 63.6% malnutrition at the end of radiotherapy. Another study by Citak et al. [34] reported that 90% of patients with head and neck cancer who received radiotherapy were well-nourished at baseline, and the rate was only 26% at the end of the treatment. In our research, the rate of nutritional risk and malnutrition raised from 4.3% to 12.8% at the onset of proton radiation to 6.4% and 27.7% at the end of the treatment (Table 2). However, the proportion of malnutrition showed no significant differences over PRT. Those changes over time seemed less obvious than that Unsal et al. [10], Hill et al. [6], and Citak et al. [34] reported.

Weight loss was one of the common symptoms of malnutrition, and may correlate to clinical outcomes. Cacicedo et al. [35] reported an average weight loss was 2.35 kg, and 65.7% of cancer patients had unintentional weight loss during radiotherapy. Another prospective study showed weight loss was present in 56% at the end of radiotherapy, which was associated with a higher risk of death in 10-yearfollow-up [36]. Weight loss has also been reported in patients undergoing proton therapy. Zhang et al. [21] reported that 58.72% of patients with head and neck cancer had weight loss at the end of proton and heavy ion radiotherapy. And for patients treated with proton beam craniospinal irradiation (p-CSI), Barney et al. [37] reported the median weight loss was 1.6% (range from 10% weight loss to 14% weight gain). Another study of medulloblastoma patients showed the median percentage of weight change was −1.2% (range, +14 to −8.4%) for p-CSI received patients and −5.8% (range, +5.8 to −17.1%) for conventional photon craniospinal irradiation (x-CSI) received patients, and less p-CSI received patients experienced >5% weight loss [17]. According to this present study, the median percentage of weight change was 0% (range, +9.2 to −5.3%), 42.6% of patients experienced weight loss during the PRT, only 1 patient had weight loss over 5%, and 57.4% of patients maintained or gained body weight, in general the weight showed stable over PRT (Tables 2 and 5). These changes were more similar to the findings in patients treated with proton therapy than those treated with conventional radiation.

The HGS test is a convenient and effective method for assessing skeletal muscle function in clinical practice. Nowadays, HGS is considered as an outcome predictor and marker of nutritional status [38, 39]. Previous studies reported reductions in HGS over anticancer treatment. Chauhan et al. [40] described that head and neck cancer patients experienced a significant decrease of 5.7 kg in HGS after 7 weeks of chemoradiotherapy. Another research similarly reported that HGS of esophageal cancer patients significantly decreased during chemoradiotherapy [9]. However, in this study, no significant reductions were observed in HGS of cancer patients over PRT (Table 4).

Anthropometric parameters are other factors that are associated with nutritional status [41]. In the present study, the average values of weight, BMI, TSF, MUAC, and MAMC were stable along the treatment (Table 5). Our results were different from the findings of many other researches. Citak et al. [34] reported a reduction in mid-arm upper circumference, and mid-arm muscle mass of head and neck cancer patients after radiotherapy. Movahed et al. [9] observed significant reductions in anthropometric parameters of esophageal cancer patients, including MUAC, fat mass percentage, and fat free mass index.

Hematological parameters including TP, ALB and HGB, are commonly used observational indicators in nutritional surveys. Those parameters can reflect patients' nutritional status but also can be affected by disease status, treatments, and metabolic status such as inflammation, infection, surgery, trauma, etc [5, 41, 42]. Nevertheless, changes in diseases and metabolic status might aggravate patients' nutritional status [5]. Previous study has shown that the levels of serum protein and albumin significantly decreased in head and neck cancer patients who were treated with radiotherapy [34]. Movahed et al. [9] observed significant reductions in the level of white blood cells, total lymphocyte count, hemoglobin, serum total protein, and albumin of esophageal cancer patients during chemoradiotherapy. In this research, we investigated TP, ALB, and HGB over PRT. We observed that the reductions were insignificant in the level of TP or ALB, and the level of HBG was even higher at the end of PRT (Table 6). And our findings differed from that reported by Citak et al. [34], and Movahed et al. [9]. However, lighter acute hematological toxicities of proton therapy have been reported. Barney et al. [37] described low rates of acute toxicity in adult patients treated with p-CSI, in their research, the median percent of hemoglobin, compared to the baseline, was 97% (range, 65 to 112%) at nadir and 103% (range, 79 to 130%) a month after proton beam radiation therapy. Brown et al. [17] reported that p-CSI received medulloblastoma patients had smaller reductions in peripheral white blood cells, hemoglobin, and platelets compared with x-CSI received patients (*p* < 0.05). Based on previous research [17, 37], our findings in hemoglobin may be explained by the reduction of toxicities of proton radiation, but more research should be conducted.

In China, proton therapy is only available in very rare hospitals. To our knowledge, this is the first study that observed the changes in the nutrition of PRT receiving cancer patients. We also acknowledge that there are limitations of this study. First, the sample size was small and may restrict the definite effect of proton radiation in the nutrition of cancer patients. And the prevalence of malnutrition varied with tumor type, stage, and location, the effect of proton radiation on different types of patients should be investigated separately. Secondly, the hematological parameters we investigated in this study are less sensitive as indicators of nutritional status. Dynamic nutrition-associated markers such as prealbumin, retinol-binding protein, transferrin, and others should be detected in our future research. Thirdly, we only investigated nutritional status during treatment, the adverse effects and the association with nutritional status should be involved, and the follow-up investigations including nutritional status and clinical outcomes are necessary to be explored in our future research. Furthermore, we did not compare the nutritional status of PRT receiving patients with those receiving conventional photon radiation therapy, and the comparison will be investigated in our future study.

In summary, the nutritional risk and nutritional status of patients undergoing PRT were investigated in this observational study. We observed that the rate of nutritional risk and malnutrition had a lighter rise from 4.3% to 12.8% up to 6.4% and 27.7% at the end of proton radiotherapy. And patients' dietary intake, HGS, anthropometric indicators, and hematological parameters showed no significant decrease over the treatment. The results of this study indicated that proton radiotherapy might have a lighter effect on the nutritional status of cancer patients. However, we are unable to definitively determine the effect due to the small number of patients, and further investigation should be evaluated in future research. Besides, we still need to pay more attention to the patients on their nutritional status along the treatment, and timely provide appropriate nutritional intervention.

## Figures and Tables

**Table 1:** Characteristics of patients.

Characteristics	Range	Median (IQR)
Age (y)	26–76	55 (38, 63)
Weight (kg)	42–99	65 (58, 78)
BMI (kg/m^2^)	19.17–36.73	24.61 (21.64, 26.44)
Hospitalization duration (day)	33–78	56 (52, 63)

Characteristics	*n*	%

Tumor site		
Head and neck	12	25.5
Intracranial	13	27.7
Lung and chest	6	12.8
Abdomen, pelvis, and others	16	34.0

Tumor stage		
I∼II	11	23.4
III∼IV	12	25.5
Other	26	51.1

Education		
Primary school or no school	7	14.9
High school	26	53.3
College or above	14	29.8

Marital status		
Married	43	91.5
Single or along	4	8.8

IQR: interquartile range, BMI: body mass index.

**Table 2:** Changes in nutritional risk and nutritional status of hospitalized patients at onset and end of PRT.

Characteristics, *n* (%)	At onset	In the end	*p* value^*∗*^
NRS 2002			1.000
<3	45 (95.7%)	44 (93.6%)	
≥3	2 (4.3%)	3 (6.4%)	
PG SGA			0.144
A (well nourished)	41 (87.2%)	34 (72.3%)	
B (moderate malnourished)	6 (12.8%)	11 (23.4%)	
C (severe malnourished)	0 (0.0%)	2 (4.3%)	
Weight change, %, median (range)		0.00% (−5.3% to 9.2%)	
Gain		15 (31.9%)	
Stable		12 (25.5%)	
Loss		20 (42.6%)	
<5%		19 (40.4%)	
≥5%		1 (2.1%)	
BMI			1.000
Underweight (<18.5 kg/m^2^)	0 (0.0%)	0 (0.0%)	
Normal weight (18.5–24.9 kg/m^2^)	24 (51.1%)	24 (51.1%)	
Overweight (25–29.9 kg/m^2^)	21 (44.7%)	21 (44.7%)	
Obese (≥30 kg/m^2^)	2 (4.2%)	2 (4.2%)	

^*∗*^Based on Fisher's exact test. PRT: proton radiotherapy, NRS 2002: nutritional risk screening 2002, PG SGA: patient generated subjective global assessment, BMI: body mass index.

**Table 3:** Changes in 24 h dietary intake of hospitalized patients at onset and end of PRT.

Variables	Onset of PRT	End of PRT	*T/Z* value	*p* value
Energy intake (kcal)^#^	1454.34 ± 204.52	1427.79 ± 263.64	−0.614	0.539
Energy intake/current weight (kcal/kg)^*∗*^	21.81 ± 3.44	21.34 ± 4.08	−1.089	0.282
Protein intake (g)^#^	64.26 ± 9.67	65.66 ± 11.43	−1.235	0.217
Protein intake/current weight (g/kg)^#^	0.96 ± 0.16	0.98 ± 0.20	−1.101	0.271

^*∗*^Analyzed by paired *t*-test. ^#^Analyzed by Wilcoxon signed rank test. PRT: proton radiotherapy.

**Table 4:** Changes in HGS of hospitalized patients at onset and end of PRT.

Variables	Onset of PRT	End of PRT	*T/χ * ^2^ value	*p* value
HGS (kg)^*∗*^	31.35 ± 10.06	30.16 ± 9.87	−1.645	0.107
LHS (*n*)^#^	6 (12.8%)	5 (10.6%)	0.103	0.748

^*∗*^Analyzed by paired *t*-test. ^#^Analyzed by Pearson's *χ*^2^ test. PRT: proton radiotherapy, HGS: hand grip strength, LHS: low handgrip strength.

**Table 5:** Changes in anthropometric parameters of hospitalized patients at onset and the end of PRT.

Variables	Onset of PRT	End of PRT	*T/Z* value	*p* value
Weight (kg)^*∗*^	68.04 ± 12.68	68.04 ± 12.42	0.000	1.000
BMI (kg/m^2^)^#^	24.57 ± 3.51	24.58 ± 3.31	−0.107	0.915
MUAC (cm)^#^	27.49 ± 2.97	27.34 ± 2.65	−0.643	0.520
MAMC (cm)^*∗*^	23.17 ± 2.69	23.06 ± 2.52	−0.519	0.606
TSF (mm)^#^	13.77 ± 5.47	13.63 ± 5.39	−0.081	0.935

^*∗*^Analyzed by paired *t*-test. ^#^Analyzed by Wilcoxon signed rank test. PRT: proton radiotherapy, BMI: body mass index, MUAC: mid-upper arm circumference, MAMC: mid-upper arm muscle circumference, TSF: triceps skinfold thickness.

**Table 6:** Changes in the hematological parameters of hospitalized patients at onset and end of PRT.

Variables	Onset of PRT (*n*)	End of PRT (*n*)	*T/Z*value	*p* value
TP (g/L)^#^	70.73 ± 6.15 (46)	71.15 ± 5.10 (47)	−0.262	0.793
ALB (g/L)^*∗*^	43.52 ± 3.53 (46)	43.61 ± 3.36 (47)	0.167	0.868
HGB (g/L)^*∗*^	134.04 ± 15.52 (47)	137.47 ± 14.45 (47)	2.231	0.031

^*∗*^Analyzed by paired *t*-test. ^#^Analyzed by Wilcoxon signed rank test. PRT: proton radiotherapy, TP: total protein, ALB: albumin, HGB: hemoglobin.

## Data Availability

The data used to support the findings of this study are included within the article.
